# LncRNA SNHG12 regulates the radiosensitivity of cervical cancer through the miR-148a/CDK1 pathway

**DOI:** 10.1186/s12935-020-01654-5

**Published:** 2020-12-01

**Authors:** Chen Wang, Shiqing Shao, Li Deng, Shelian Wang, Yongyan Zhang

**Affiliations:** 1 Department of Obstetrics and Gynecology, Huaihe Hospital of Henan University, No.8 Baogonghu North Road, Kaifeng, 475000 Henan China; 2 Department of Obstetrics and Gynecology, The Second Affiliated Hospital of Guangxi Medical University, Nanning, Guangxi China

**Keywords:** Cervical cancer, Radiosensitivity, SNHG12, miR-148a, CDK1

## Abstract

**Background:**

Radiation resistance is a major obstacle to the prognosis of cervical cancer (CC) patients. Many studies have confirmed that long non-coding RNAs (lncRNAs) are involved in the regulation of radiosensitivity of cancers. However, whether small nucleolar RNA host gene 12 (SNHG12) regulates the radiosensitivity of CC remains unknown.

**Methods:**

Quantitative real-time polymerase chain reaction was used to measure the expression levels of SNHG12 and microRNA-148a (miR-148a). The radiosensitivity of cells was evaluated by clonogenic assay. Flow cytometry and caspase-3 activity assay were performed to assess the apoptosis ability and cell cycle distribution of cells. Besides, dual-luciferase reporter and RNA immunoprecipitation assay were used to verify the interaction between miR-148a and SNHG12 or cyclin-dependent kinase 1 (CDK1). Also, the protein levels of CDK1, CCND1 and γ-H2AX were detected by western blot analysis. Furthermore, in vivo experiments were conducted to verify the effect of SNHG12 on CC tumor growth. Ki-67 and TUNEL staining were employed to evaluate the proliferation and apoptosis rates in vivo. The hematoxylin and eosin (HE) staining were employed to evaluate the tumor cell morphology.

**Results:**

SNHG12 was upregulated in CC tissues and cells, and its knockdown improved the radiosensitivity by promoting the radiation-induced apoptosis and cell cycle arrest of CC cells. Also, miR-148a could be sponged by SNHG12 and could target CDK1. MiR-148a inhibitor or CDK1 overexpression could invert the promotion effect of silenced-SNHG12 on CC radiosensitivity. Meanwhile, SNHG12 interference reduced the tumor growth of CC, increased miR-148a expression, and inhibited CDK1 level in vivo.

**Conclusion:**

LncRNA SNHG12 promoted CDK1 expression to regulate the sensitivity of CC cells to radiation through sponging miR-148a, indicating that SNHG12 could be used as a potential biomarker to treat the radiotherapy resistance of CC patients.

## Background

Cervical cancer (CC) is one of the most common malignant tumors in women, which poses a severe threat to women’s health [1, 2]. CC can be eliminated through early prevention and treatment, and radiotherapy is the main mean of CC treatment [3, 4]. However, the emergence of radiotherapy resistance seriously hinders the treatment process of CC, resulting in poor efficacy of CC patients [5, 6]. Thus, it is particularly important to search for biomarkers related to radiosensitivity for the study of CC treatment.

Long non-coding RNAs (lncRNAs) are non-coding protein RNAs with a length of over 200 nucleotides (nts), which have been proved to be involved in the regulation of many diseases, including cancer [7, 8]. In recent years, researchers have found that lncRNAs also take part in cancer radiotherapy resistance. Liu et al*.* reported that knockdown of lncRNA FAM201A improved the radiosensitivity of non-small-cell lung cancer (NSCLC) [9]. Besides, Zhao et al*.* revealed that lncRNA LINC00958 silencing could enhance radiosensitivity in CC [10]. Small nucleolar RNA host gene 12 (SNHG12) is a lncRNA widely expressed in various cancers, including gastric cancer and laryngeal cancer [11, 12]. Studies have shown that SNHG12 is highly expressed in CC, and is related to the metastasis of CC [13]. Despite this, it is unclear whether SNHG12 affects the radiosensitivity of CC.

As is known to all, microRNAs (miRNAs) are key regulators of gene expression [14]. Researches have shown that lncRNAs can bind to miRNAs as the competitive endogenous RNAs (ceRNAs) and participate in the regulation of gene expression [15]. MiR-148a can be adsorbed by many lncRNAs to involve in regulating cancer progressions, such as prostate cancer and osteosarcoma [16, 17]. Many studies have indicated that miR-148a is lower expressed in CC and is related to the progression of CC [18, 19]. Cyclin-dependent kinase 1 (CDK1), a member of the CDKs family, is an important regulator of the cell cycle. Previous studies showed that CDK1 is highly expressed in many cancers, and can act as a target gene to regulate cancer progression [20, 21]. Raghavan et al*.* revealed that CDK1 inhibitor could enhance the radiosensitivity of NSCLC [22]. Additionally, it was reported that CDK1 could promote CC progression [23]. Therefore, the study of miR-148a and CDK1 will help us better understand the molecular mechanism influencing the radiosensitivity of CC.

The purpose of this study was to investigate the role of SNHG12 in CC radiotherapy, and to clarify its potential molecular mechanism through bioinformatics analysis and experimental verification. In our study, we found that SNHG12 was differentially expressed in CC tissues before and after radiotherapy, so it was speculated that SNHG12 expression might be related to the radiosensitivity of CC. Further tests confirmed that the absence of SNHG12 could enhance the radiosensitivity of CC. In terms of mechanism, we confirmed that SNHG12 could regulate the expression of CDK1 by targeting miR-148a to mediate CC radiosensitivity, which might provide a new strategy for us to improve CC radiosensitivity.

## Materials and methods

### Tissue samples collection

39 CC patients who had not received radiotherapy were recruited from Huaihe Hospital of Henan University, and their CC tissues (before radiotherapy) and adjacent normal tissues were taken and stored at – 80 °C. After radiotherapy, CC tissues (after radiotherapy) were taken from 39 CC patients. All patients signed informed consents. This experiment was approved by the Ethics Committee of Huaihe Hospital of Henan University.

### Cell culture

Human CC cell lines (SiHa and Hela) and normal cervical epithelial cell line (Ect1/E6E7) were obtained from American Type Culture Collection (ATCC, Manassas, VA, USA) and cultured in Dulbecco’s modified Eagle’s medium (DMEM; Gibco, Carlsbad, CA, USA) containing 10% fetal bovine serum (FBS; HyClone, Logan, UT, USA), 100 U/mL penicillin and 100 μg/mL streptomycin (Solarbio, Beijing, China) at 37 °C with 5% CO_2_.

### Quantitative real-time polymerase chain reaction (qRT-PCR)

Total RNA was isolated using Trizol reagent (Invitrogen, Carlsbad, CA, USA). PrimeScript RT Master Mix Perfect Real-Time (Takara, Dalian, China) was used to reverse-transcribed RNA into complementary DNA (cDNA). SYBR Green Master Mix (Vazyme, Nanjing, China) was used to perform qRT-PCR. U6 and β-actin were used as endogenous controls. Data analysis was calculated using the 2^−∆∆Ct^ method. All primers were designed as following: SNHG12, F 5′-GGTGCTCCAGGCAATAACT-3′, R 5′-CTCCCATACAGTCCGAACAT-3′; miR-148a, F 5′-ACACTCCAGCTGGGTCAGTGCACTACAGAA-3′, R 5′-TGGTGTCGTGGAGTCG-3′; CDK1, F 5′-TGAGGTAGTAACACTCTGGTA-3′, R 5′-ATGCTAGGCTTCCTGGTT-3′; U6, F 5′-CTCGCTTCGGCAGCACATA-3′, R 5′-CGAATTTGCGTGTCATCCT-3′; β-actin, F 5′-CTCCATCCTGGCCTCGCTGT-3′, R 5′-GCTGTCACCTTCACCGTTCC-3’.

### Cell transfection

SNHG12 small interfering RNA and overexpression plasmid (si-SNHG12 and SNHG12) or their negative controls (si-con and pcDNA), miR-148a mimic and inhibitor (miR-148a and anti-miR-148a) or their negative controls (miR-con and anti-miR-con), CDK1 overexpression plasmid (CDK1) and its negative control (pcDNA) were designed and synthesized by GenePharma (Shanghai, China). Lentiviral short hairpin RNA targeting SNHG12 (sh-SNHG12) and its negative control (sh-con) were constructed by Genechem (Shanghai, China). Cells were transfected with indicated plasmids using Lipofectamine 3000 (Invitrogen).

### Clonogenic assay

SiHa and Hela cells (1000 cell per plate) were seeded into 6-well plates and irradiated with X-ray at different radiation doses (0 Gy, 2 Gy, 4 Gy, 6 Gy and 8 Gy). After incubation for 2 weeks, the colonies formed by the cells were fixed with methanol and stained with crystal violet. Then, the number of colonies (> 50 cells) was counted, and the survival fraction was calculated. The survival fraction of 0 Gy was considered as the control and all data were normalized to the survival fraction of 0 Gy.

### Flow cytometry

SiHa and Hela cells (1 × 10^6^) were seeded in 6 well-plates and were exposed to 0 Gy or 2 Gy of radiation. After transfection for 48 h, cells were harvested and centrifuged to remove the supernatant. For cell apoptosis assay, the cells were re-suspended with binding buffer and stained with Annexin V-fluorescein isothiocyanate (FITC) and propidium iodide (PI) (all from BestBio, Shanghai, China). The apoptosis of cells was evaluated by the flow cytometer (Beckman Coulter, San Jose, CA, USA). For cell cycle distribution assay, the cells were washed with precooled PBS and fixed with 75% ethanol. Then, the cells were washed with PBS and stained with PI and RNase A (Beyotime, Shanghai, China). The cell cycle distribution of cells was determined using the flow cytometer.

### Caspase-3 activity assay

After radiation treatment and transfection for 48 h, SiHa and Hela cells (1 × 10^5^) were harvested, centrifuged, and lysed with lysis buffer (Beyotime) for 15 min. After centrifugation, the cell lysates were collected and caspase-3 activity was detected with the Caspase-3 Activity Assay Kit (Beyotime).

### Dual-luciferase reporter assay

SNHG12 fragment containing predicted miR-148a binding sites and mutant binding sites were cloned into pGL3-control vector (Promega, Madison, WI, USA), forming the SNHG12-WT and SNHG12-MUT reporter vectors. Similarly, the CDK1-WT and CDK1-MUT reporter vectors were built in the same way. Lipofectamine 3000 (Invitrogen) was used to co-transfect the reporter vectors with miR-148a mimic and inhibitor or their negative controls into SiHa and Hela cells. After 48 h, the luciferase activities of cells were detected by the Dual-Luciferase Reporter Assay System (Promega).

### RNA immunoprecipitation (RIP) assay

SiHa and Hela cells were lysed with RIP lysis buffer (Millipore, Billerica, MA, USA) and incubated with immunoglobulin G (IgG) antibody (Anti-IgG) and argonaute2 (Ago2) antibody (Anti-Ago2) coated on magnetic beads (Millipore) overnight at 4 °C. Part of the cell lysate was used as a negative control and named as Input. After the immunoprecipitates were purified, the enrichments of SNHG12, miR-148a and CDK1 were detected by qRT-PCR.

### Western blot (WB) analysis

Protein was extracted using RIPA buffer (Beyotime). Then, cell lysates were separated by sodium dodecyl sulfate-polyacrylamide gel electrophoresis (SDS-PAGE) gel and transferred onto polyvinylidene fluoride (PVDF) membranes (Millipore). After blocking with non-fat milk for 2 h, the membranes were incubated with primary antibodies CDK1 (1:500, BA0027-2, Boster, Wuhan, China), CCND1 (1:2000, PB0403, Boster), γ-H2AX (1:1000, AF5836, Beyotime) and β-actin (1:5000, BA2305, Boster) overnight at 4 °C, followed by incubating with secondary antibody (1:10,000, BA1056, Boster) for 1 h. Immunoreactive bands were visualized using enhanced chemiluminescence reagent (Millipore).

### In vivo experiments

Eighteen BALB/c-nude mice (5-week-old, male, Vital River, Beijing, China) were randomly divided into three groups (n = 6 per group). Hela cells stably transfected with sh-SNHG12 or sh-con, as well as un-transfected Hela cells (Empty), were injected into nude mice. Tumor length and width were recorded weekly, and tumor volume was calculated using length × width^2^/2 method. The mice were sacrificed after 5 weeks, and the tumors were taken for weight determination and further experimental analysis. All animal experiments were approved by the Animal Research Committee of Huaihe Hospital of Henan University.

### Ki-67 and TUNEL staining

Mice tumor tissues were taken for paraffin sectioning, and then stained with Ki-67 Immunohistochemical Kit and TUNEL Assay Kit (Yanjinbio, Shanghai, China) according to the manufacturer’s agreement.

### Hematoxylin and eosin (HE) staining

The tumor tissues of mice were paraffin sectioned and dewaxed with xylene and alcohol. The samples were then dehydrated and sealed after being stained with hematoxylin and eosin. Finally, cell morphology was observed under a microscope.

### Statistical analysis

Data were presented as mean ± standard deviation (SD) and statistically analyzed by Student’s *t*-test (for two groups) and one-way analysis of variance followed by Tukey post-hoc test (for multiple groups). Statistical analysis was performed using GraphPad Prism5.0 software (GraphPad Software, San Diego, CA, USA). *P* < 0.05 was defined as statistically significant.

## Results

### The SNHG12 expression in CC tissues and cells

Firstly, qRT-PCR was performed to detect the expression of SNHG12 in CC tissues and cells. As shown in Fig. 1a, SNHG12 level was markedly improved in CC tissues (before radiotherapy) compared with adjacent normal tissues. Surprisingly, SNHG12 expression in CC tissues after radiotherapy was remarkably lower than that before radiotherapy. Furthermore, the correlation between SNHG12 expression and the clinicopathologic features of CC patients showed that high SNHG12 expression was positively correlated with the tumor size and TNM stage of CC patients (*P* < 0.05, Table 1). Besides, compared to the Ect1/E6E7 cells, the expression of SNHG12 was also increased in SiHa and Hela cells (Fig. 1b). Hence, these results suggested that SNHG12 might be related to the radiosensitivity of CC.

**Fig. 1:** The expression of SNHG12 in CC tissues and cells. **a** The expression of SNHG12 was detected by qRT-PCR in adjacent normal tissues and CC tissues (before and after radiotherapy). **b** QRT-PCR was used to measure SNHG12 expression in CC cells (SiHa and Hela) and human normal cervical epithelial cells (Ect1/E6E7). *P < 0.05

**Table 1:** Correlation between the clinicopathologic features of CC patients and the expression of SNHG12 or miR-148a

Clinicopathologic features	Relative SNHG12 level		*P* value	Relative miR-148a level		*P* value
	High (%)	Low (%)		Low (%)	High (%)	
Age (years)			> 0.05			> 0.05
≥ 50	12 (57.1)	9 (42.9)		13 (61.9)	8 (30.1)	
< 50	9 (50)	9 (50)		10 (55.6)	8 (44.4)	
Tumor size (cm)			< 0.05			< 0.05
≥ 5	11 (68.8)	5 (31.2)		10 (62.5)	6 (37.5)	
< 5	10 (43.5)	13 (56.5)		13 (56.5)	10 (43.5)	
TNM stage			< 0.05			< 0.05
I + II	9 (39.1)	14 (60.9)		6 (26.1)	17 (73.9)	
III + IV	12 (75.0)	4 (25.0)		17 (65.4)	9 (34.6)	
Lymphatic metastasis			> 0.05			> 0.05
No	15(60.0)	10 (40.0)		14 (60.9)	9 (39.1)	
Yes	6 (42.9)	8 (57.1)		9 (56.3)	7 (43.7)	

### Knockdown of SNHG12 improved radiosensitivity through promoting radiation-induced apoptosis and cell cycle arrest in CC cells

To investigate the effect of SNHG12 on regulating the radiosensitivity of CC, we transfected with si-SNHG12 and si-con into SiHa and Hela cells. Clonogenic assay showed that silencing of SNHG12 significantly reduced the survival fractions of SiHa and Hela cells compared with the si-con group (Fig. 2a, b). Further, flow cytometry results revealed that apoptosis was increased in the presence of 2 Gy radiation, and was even more serious after silenced-SNHG16 in SiHa and Hela cells (Fig. 2c, d). Meanwhile, we also tested the activity of caspase-3, and the results confirmed that radiation could increase the apoptosis rate of SiHa and Hela cells and the apoptosis rate was even higher after SNHG12 knockdown, while the addition of caspase inhibitor zvad-fmk could markedly reverse the promoting effect of SNHG12 knockdown on the apoptosis of CC cells to restrain apoptosis (Fig. 2e, f). Additionally, we also measured the cell cycle distribution in SiHa and Hela cells. As shown in Fig. 2g, h, we found that radiation could induce cell arrest in G0–G1 phase and inhibit the number of cells in S phase, while SNHG12 silencing also could exacerbate this process, indicating that SNHG12 knockdown restrained the cell cycle in CC cells. By detecting the protein expression of CCND1, we uncovered that silenced SNHG12 could accelerate the suppression effect of radiation on the CCND1 protein expression in SiHa and Hela cells (Fig. 2i, j). All data indicated that the effect of SNHG12 on radiosensitivity in CC was mainly achieved by regulating radiation-induced apoptosis and cell cycle arrest.

**Fig. 2:** Effects of SNHG12 knockdown on radiosensitivity in CC cells. SiHa and Hela cells were transfected with si-SNHG12 or si-con. **a**, **b** Clonogenic assay was performed to assess the survival fractions of SiHa and Hela cells. **c**, **d** The apoptosis of SiHa and Hela cells treated with different doses of radiation (0 Gy and 2 Gy) was determined by flow cytometry. **e**, **f** The caspase-3 activity of SiHa and Hela cells treated with different doses of radiation (0 Gy and 2 Gy) was detected by Caspase-3 Activity Assay Kit. **g**, **h** Flow cytometry was used to examine the cell cycle distribution in SiHa and Hela cells treated with different doses of radiation (0 Gy and 2 Gy). **i**, **j** WB analysis was performed to measure the protein expression of CCND1 in SiHa and Hela cells treated with different doses of radiation (0 Gy and 2 Gy). *P < 0.05

### SNHG12 directly sponged miR-148a

To explore the mechanism of SNHG12 in SiHa and Hela cells, we predicted the potential target miRNAs of SNHG12 using the DIANA TOOLS (https://diana.imis.athena-innovation.gr/DianaTools/index.php?r=site/page&view=software). As shown in Fig. 3a, miR-148a had complementary sites with SNHG12. In order to verify this targeting relationship between them, we conducted the dual-luciferase reporter assay. The results revealed that miR-148a overexpression markedly decreased the luciferase activity of SNHG12-WT vector, while miR-148a inhibitor significantly increased the luciferase activity of SNHG12-WT vector, but both had no effect on the luciferase activity of SNHG12-MUT vector in SiHa and Hela cells (Fig. 3b, c). Furthermore, RIP assay results showed that in SiHa and Hela cells, SNHG12 and miR-148a were markedly enriched in Anti-Ago2, which once again proved that SNHG12 might be related to miR-148a (Fig. 3d, e). In addition, we transfected SNHG12 overexpression plasmid and si-SNHG12 into SiHa and Hela cells and found that miR-148a expression was inhibited by SNHG12 overexpression, while promoted by SNHG12 silencing (Fig. 3f, g). Therefore, the above results confirmed that miR-148a was sponged by SNHG12 in CC cells.

**Fig. 3:** SNHG12 acted as a sponge of miR-148a. **a** The sequences of SNHG12 containing the miR-148a binding sites and mutant binding sites were shown. **b**, **c** Dual-luciferase reporter assay was used to verify the binding of SNHG12 in miR-148a. **d**, **e** RIP assay was performed to determine the enrichment of SNHG12 and miR-148a in Anti-IgG, Anti-Ago2 and Input. **f**, **g** The effect of SNHG12 expression on the expression of miR-148a in SiHa and Hela cells was detected by qRT-PCR. *P < 0.05

### CDK1 was a target of miR-148a

Similarly, DIANA TOOLS (https://diana.imis.athena-innovation.gr/DianaTools/index.php?r=site/page&view=software) also was used to predict the target gene of miR-148a and the results showed that CDK1 3′UTR had binding sites of miR-148a (Fig. 4a). Dual-luciferase reporter assay results indicated that the luciferase activity of CDK1-WT vector was inhibited by miR-148a overexpression, while improved by miR-148a inhibitor in SiHa and Hela cells. However, miR-148a mimic and inhibitor did not affect the luciferase activity of CDK1-MUT vector in SiHa and Hela cells (Fig. 4b, c). Moreover, Anti-Ago2 precipitated a large amount of CDK1 and miR-148a in SiHa and Hela cells compared with Anti-IgG (Fig. 4d, e). Also, we investigated the effect of miR-148a expression on CDK1 level in SiHa and Hela cells. Through detecting the protein expression of CDK1, we discovered that the level of CDK1 was hindered by miR-148a overexpression, while promoted by miR-148a knockdown in SiHa and Hela cells (Fig. 4f, g). These results suggested that miR-148a targeted CDK1 in CC cells.

**Fig. 4:** CDK1 was targeted by miR-148a. **a** The sequences of miR-148a containing the CDK1 3′UTR binding sites and mutant binding sites were shown. **b**, **c** The binding of miR-148a in 3′UTR of CDK1 was verified by dual-luciferase reporter assay. **d**, **e** The enrichments of CDK1 and miR-148a in Anti-IgG, Anti-Ago2 and Input were detected by RIP assay. **f**, **g** WB analysis was used to detect the effect of miR-148a expression on the protein level of CDK1 in SiHa and Hela cells. *P < 0.05

### SNHG12 regulated CDK1 expression by sponging miR-148a

Through the detection of miR-148a expression in CC tissues, we discovered that the expression of miR-148a in CC tissues was lower than that in adjacent normal tissues (Fig. 5a). Besides, by analyzing the correlation between miR-148a expression and the clinicopathologic features of CC patients, we uncovered that low miR-148a expression also was positively correlated with the tumor size and TNM stage of CC patients (*P* < 0.05, Table 1). In addition, we detected the expression of miR-148a and CDK1 in CC cells. QRT-PCR results determined that miR-148a expression was remarkably downregulated in SiHa and Hela cells compared with Ect1/E6E7 cells (Fig. 5b). However, CDK1 level was markedly higher in SiHa and Hela cells than that in Ect1/E6E7 cells (Fig. 5c). To confirm the regulatory effect of SNHG12 on the expression of miR-148a and CDK1, we co-transfected SNHG12 overexpression plasmid and miR-148a mimic or si-SNHG12 and miR-148a inhibitor into SiHa and Hela cells. By detecting the expression of miR-148a, we found that miR-148a overexpression could reverse the inhibitory effect of SNHG12 overexpression on miR-148a expression in SiHa and Hela cells, and likewise, miR-148a inhibitor could invert the promoting effect of SNHG12 knockdown on miR-148a expression (Fig. 5d, e). Moreover, the protein level of CDK1 was tested by WB analysis. As shown in Fig. 5f, SNHG12 overexpression promoted the expression of CDK1 in SiHa and Hela cells, while miR-148a overexpression reversed this effect. Besides, silenced-SNHG12 also impeded CDK1 expression in SiHa and Hela cells, whereas this effect also could be recovered by miR-148a inhibitor (Fig. 5g). The above results verified that miR-148a and CDK1 expression levels were regulated by SNHG12.

**Fig. 5:** Effects of SNHG12 expression on the expression levels of miR-148a and CDK1. **a** QRT-PCR was used to determine miR-148a expression in CC tissues and adjacent normal tissues. **b** The expression of miR-148a in CC cells (SiHa and Hela) and Ect1/E6E7 cells was detected by qRT-PCR. **c** The protein level of CDK1 in CC cells (SiHa and Hela) and Ect1/E6E7 cells was measured by WB analysis. **d**, **e** The expression of miR-148a was determined by qRT-PCR in SiHa and Hela cells treated with SNHG12 overexpression plasmid and miR-148a mimic or si-SNHG12 and anti-miR-148a. **f**, **g** WB analysis was used to detect the protein level of CDK1 in SiHa and Hela cells treated with SNHG12 overexpression plasmid and miR-148a mimic or si-SNHG12 and anti-miR-148a. *P < 0.05

### MiR-148a inhibitor and CDK1 overexpression could reverse the effect of SNHG12 knockdown on radiosensitivity in CC cells

To clarify the role of miR-148a and CDK1 in CC cells, we co-transfected si-SNHG12 and anti-miR-148a or CDK1 overexpression plasmid into SiHa and Hela cells. Clonogenic assay results indicated that compared with the corresponding negative controls, both miR-148a inhibitor and CDK1 overexpression could recover the inhibitory effect of SNHG12 silencing on the survival fractions of SiHa and Hela cells (Fig. 6a, b). Through the flow cytometry and caspase-3 activity detection, we also confirmed that the promotion effect of silenced-SHNG12 on cell apoptosis could also be reversed by miR-148a inhibitor and CDK1 overexpression in 2 Gy radiation treatment of SiHa and Hela cells (Fig. 6c–f). In addition, the results of cell cycle distribution assay revealed that miR-148a inhibitor and CDK1 overexpression also could invert the suppression effect of SNHG12 knockdown on the percentage of SiHa and Hela cells in S phase under 2 Gy radiation (Fig. 6g, h). Furthermore, the protein expression of CCND1 inhibited by SNHG12 silencing also could be reversed by miR-148a inhibitor and CDK1 overexpression in SiHa and Hela cells (Fig. 6i, j). Therefore, our data suggested that SNHG12 regulated the radiosensitivity of CC cells by the miR-148a/CDK1 axis.

**Fig. 6:** Effects of miR-148a inhibitor and CDK1 overexpression on radiosensitivity, apoptosis and cell cycle in CC cells. SiHa and Hela cells were transfected with si-SNHG12 and anti-miR-148a or CDK1 overexpression plasmid. **a**, **b** The survival fractions of SiHa and Hela cells were assessed by clonogenic assay. **c**, **d** Flow cytometry was used to determine the apoptosis of SiHa and Hela cells treated with 2 Gy radiation. **e**, **f** Caspase-3 Activity Assay Kit was used to detect the caspase-3 activity of SiHa and Hela cells treated with 2 Gy radiation. **g**, **h** The cell cycle distribution in SiHa and Hela cells treated with 2 Gy radiation was determined using flow cytometry. **i**, **j** The protein expression of CCND1 in SiHa and Hela cells treated with 2 Gy radiation was tested by WB analysis. *P < 0.05

### Interference of SNHG12 reduced the tumor growth of CC in vivo

To further verify the function of SNHG12 in CC, we constructed the mice xenograft models. After 5 weeks of detection, we found that the tumor volume of mice in the SNHG12 knockdown group was significantly smaller than that of the control group (Fig. 7a). Also, the tumor weight of mice was markedly lower in the SNHG12 knockdown group than in the control group (Fig. 7b). At the same time, we detected the expression levels of SNHG12, miR-148a and CDK1 in the tumor. QRT-PCR results indicated that compared with the control group, SNHG12 expression was remarkably reduced, while miR-148a was markedly improved in the SNHG12 knockdown group (Fig. 7c, d). Besides, WB analysis revealed that CDK1 level was significantly inhibited in the SNHG12 knockdown group (Fig. 7e). Additionally, Ki-67 and TUNEL staining results confirmed that compared to the control group, the Ki-67 positive rate was obviously decreased, while the apoptosis rate was markedly enhanced in the sh-SNHG12 group (Fig. 7f). Furthermore, the HE staining results were shown in Fig. 7g. All data confirmed that SNHG12 played a tumor-promoter role in CC.

**Fig. 7:** Effects of SNHG12 knockdown on the tumor growth of CC in vivo. The CC mice xenograft models were constructed by injecting sh-con or sh-SNHG12 transfected Hela cells and un-transfected Hela cells (Empty) into nude mice. **a** Tumor volume was calculated at the indicated time point. **b** Tumor weight was measured in mice. **c**, **d** The expression levels of SNHG12 and miR-148a were detected by qRT-PCR. **e** The protein level of CDK1 was evaluated by WB analysis. **f** The results of Ki-67 and TUNEL staining were presented. **g** The pictures of HE staining was exhibited.*P < 0.05

## Discussion

Since the sensitivity of cancer cells to radiotherapy is directly related to the prognosis of patients [5, 6], the exploration of biomarkers affecting radiosensitivity has become a hot topic in cancer research. The expression of lncRNAs is closely related to the development of cancers and involved in the regulation of radiosensitivity of various cancer cells, so the study of lncRNAs is of great clinical value. In CC, lncRNA GAS5, HOTAIR and LINC00958 have been proved to be associated with the radiosensitivity of CC cells [10, 24, 25]. Here, we found that SNHG12 was upregulated in CC, which was consistent with the results of Jin et al*.* [13]. Also, SNHG12 expression was markedly decreased in CC tissues after radiation and was reduced in CC cells under radiation in a dose-dependent manner. Therefore, we speculated that SNHG12 might play an important role in the radiosensitivity of CC. Additionally, the correlation between SNHG12 expression and tumor size and TNM stage in CC patients indicated that expression of SNHG12 was closely related to the malignancy of CC patients’ tumors. Further experiments showed that silenced-SNHG12 remarkably enhanced the sensitivity of CC cells to radiation through accelerating radiation-induced apoptosis and cell cycle arrest. Due to changes in the cell cycle, we explored whether si-SNHG12 might mediate DNA damage repair. By testing the expression of DNA damage repair marker gene γ-H2AX in SiHa cells, and found that si-SNHG12 could promote the expression of γ-H2AX (Additional file 1: Fig. S1). Therefore, we speculated that SNHG12 might participate in the regulation of CC cell radiosensitivity by regulating DNA damage repair. Of course, this needs further experimental verification. In addition, the results of in vivo experiments showed that knockdown of SNHG12 could inhibit the tumor growth of CC and thus achieving the purpose of anti-cancer in CC.

There is much evidence that miRNAs are directly involved in radiation resistance. For instance, miR-20a-5p could promote radio-resistance in nasopharyngeal cancer [26], while miR-9 could enhance radiosensitivity in NSCLC [27]. In our study, we uncovered that miR-148a could bind to SNHG12 in a complementary manner. Besides, consistent with the study of Zhang et al*.* [18], we found that miR-148a was downregulated in CC tissues and cells. Further, we also discovered that miR-148a expression was negatively related to the tumor size and TNM stage of CC patients. Also, miR-148a expression was regulated by SNHG12 in vitro and in vivo, which once again confirmed that miR-148a could be targeted by SNHG12. In addition, functional analysis showed that miR-148a inhibitor could reverse the promoting effect of SNHG12 knockdown on the radiosensitivity of CC cells, indicating that miR-148a was a key regulatory factor of SNHG12 in CC.

In view of the mechanism of miRNA, we predicted the potential target mRNA of miR-148a and confirmed that CDK1 was a target of miR-148a. Li et al*.* reported that CDK1 was overexpressed in CC [23], which was verified again in this study. Studies on the sensitivity of CDK1 to cancer radiotherapy have been reported previously [22, 28]. Studies have shown that the correlation between CDK1 and radiosensitivity may be due to CDK1-mediated DNA damage and repair [29, 30]. Here, we also determined that SNHG12 could regulate CDK1 protein level in vitro and in vivo. Further analysis manifested that CDK1 overexpression inverted the acceleration effect of silenced-SNHG12 on the radiosensitivity of CC cells, which confirmed the inhibitory effect of CDK1 on cell radiosensitivity and clarified that CDK1 could participate in the regulation of SNHG12 on CC radiosensitivity.

At present, there are few reports on the sensitivity of SNHG12 in radiotherapy. Our research has provided evidence that SNHG12 regulates the sensitivity of CC radiotherapy, which has pioneered the relationship between SNHG12 and cancer radiosensitivity and has important clinical significance. Furthermore, the proposed SNHG12/miR-148a/CDK1 axis also provides a new regulatory network for exploring the molecular mechanism of SNHG12, and also provides a new target for improving the radiosensitivity of CC. However, there are some limitations in this study. In animal experiments, we only tested the expression of SNHG12 in subcutaneously transplanted tumors, but did not detect the clonality of the cells or distinguish the cellular composition of the transplanted tumors. This is not rigorous, we will continue to improve our experimental design in future experiments.

## Conclusion

In summary, this study demonstrated that knockdown of SNHG12 contributed to the development of radiosensitivity in CC. Also, we illustrated that SNHG12 mediated the regulation of the sensitivity of CC cells to radiation through adsorbing miR-148a to promote CDK1 expression. Our results provided a theoretical basis for how to promote the radiosensitivity of CC to improve the prognosis of CC patients.

## Supplementary information

**Additional file 1: Fig. S1.** Effect of SNHG12 silencing on γ-H2AX expression. WB analysis was used to determine the protein expression of γ-H2AX in SiHa cells treated with different doses of radiation (0 Gy and 2 Gy).

## Data Availability

The datasets used and/or analysed during the current study are available from the corresponding author on reasonable request.

## Abbreviations

CC: Cervical cancer
SNHG12: Small nucleolar RNA host gene 12
qRT-PCR: Quantitative real-time polymerase chain reaction
RIP: RNA immunoprecipitation
CDK1: Cyclin-dependent kinase 1
WB: Western blot
NSCLC: Non-small-cell lung cancer
ATCC: American Type Culture Collection
FITC: Fluorescein isothiocyanate
PI: Propidium iodide
PVDF: Polyvinylidene fluoride
